The article "Salvianolic Acid A Suppresses DNCB-Induced Atopic Dermatitis-Like Symptoms in BALB/c Mice" was published in 2021. Journal: Evid Based Complement Alternat Med.

# Salvianolic Acid A Suppresses DNCB-Induced Atopic Dermatitis-Like Symptoms in BALB/c Mice

**DOI:** 10.1155/2021/7902592

**Published:** 2021-10-14

**Authors:** Wi-Jin Jeon, Ju-Hyun Lee, Jung-Eun Lee, So-Eun Son, Fumikazu Okajima, Ki Wung Chung, Dong-Soon Im

**Affiliations:** ^1^College of Pharmacy, Pusan National University, Busan 46241, Republic of Korea; ^2^Department of Biomedical and Pharmaceutical Sciences, Graduate School, Kyung Hee University, Seoul 02446, Republic of Korea; ^3^Department of Biomedical and Faculty of Pharmaceutical Sciences, Aomori University, Aomori 030-0943, Japan

## Abstract

Prevalence of atopic dermatitis (AD), a chronic, pruritic, and relapsing inflammatory skin disorder, is growing. Because available therapeutics is limited, immune regulators from natural resources could be helpful for treating AD symptoms. The root of *Salvia miltiorrhiza* Bunge (Lamiaceae) has been studied for the treatment of inflammatory diseases, including dermatologic disorders in Korea. This study examined the effect of salvianolic acid A on AD-like symptoms. Sensitization on the dorsal skin and repeated application on the ears with 2,4-dinitrochlorobenzene (DNCB) were performed in BALB/c mice to induce AD-like skin lesions. After induction of atopic dermatitis, salvianolic acid A (5 and 10 mg/kg) or dexamethasone (10 mg/kg) were administrated via intraperitoneal injection for 3 weeks. Salvianolic acid A suppressed DNCB-induced AD-like symptoms like ear skin hypertrophy and decreased mast cell infiltration into skin lesions. Salvianolic acid A not only reduced DNCB-induced increase of serum IgE but also lowered levels of the Th2 cytokines (IL-4 and IL-13), Th1 cytokine (interferon-*γ*), and Th17 cytokine (IL-17A). Furthermore, salvianolic acid A blocked DNCB-induced lymph node enlargement. In summary, these results suggest that salvianolic acid A might have a therapeutic potential for the treatment of AD.

## 1. Introduction

Atopic dermatitis (AD) is a chronic inflammatory skin disease characterized by eczematous plaques and intense pruritus [1]. AD is more common in children and infants up to 20% [2]. Chronic, pruritic, and relapsing eczematous skin lesions and elevated immunoglobulin E (IgE) levels in serum are the clinical symptoms of AD [1]. T-helper 2 (Th2) cells play major roles in pathogenesis of AD by producing IL-4, IL-5, and IL-13 [3, 4]. Although Th2 cells are important in the acute phase of AD, in the chronic phase, Th17 and Th1 cells are also contributing to the AD development by producing IL-17 and interferon (IFN)-*γ* [5–7]. Although corticosteroids have been widely used in children for many years, adverse effects of topical corticosteroids are accompanied such as acne, atrophy, perioral dermatitis, rosacea, striae, and purpura [8, 9]. Therefore, a great unmet medical need is to develop novel and effective therapeutics for AD.

The article "Salvianolic Acid A Suppresses DNCB-Induced Atopic Dermatitis-Like Symptoms in BALB/c Mice" was published in 2021. Journal: Evid Based Complement Alternat Med.

Human AD-like skin lesions are induced by several animal models including models induced by epicutaneous exposure to sensitizers [10]. A cytotoxic and electrophilic benzene derivative, 2,4-dinitrochlorobenzene (DNCB), was reported to induce stable clinical AD-like skin diseases in BALB/c mice [11–13]. Histological studies have shown hyperplasia and mast cells accumulation in the skin [10, 14]. BALB/c mice also shoed increased levels of serum IgE [10, 15] and T cell-mediated immune responses in the DNCB-induced pathogenesis [16, 17].

The root of *Salvia miltiorrhiza* Bunge (Lamiaceae), also known as Dan Shen, has been used in Korea, China, and Japan traditionally for the treatment of inflammatory diseases, including dermatologic disorders. *S. miltiorrhiza* is a common Chinese herb used to treat psoriasis, another skin disorder with a chronic inflammatory pathogenesis [18, 19]. Salvianolic acid B, the abundant active phytocomponent of *S. miltiorrhiza*, has shown anti-inflammatory and antioxidant effects [20, 21]. In fact, salvianolic acid B ameliorated psoriasis-like dermatitis symptoms induced by imiquimod in mice [22, 23]. The aqueous extract of Radix Salviae inhibited antidinitrophenyl immunoglobulin E (IgE)-induced passive cutaneous anaphylaxis by 72.7% and inhibited histamine release from rat peritoneal mast cells in a concentration-dependent manner [24]. Tanshinones, another group of active components isolated from *S. miltiorrhiza*, inhibited passive cutaneous anaphylaxis reaction in mice [25]. However, effects of salvianolic acid A (Sal A) have not been studied in skin disorders such as AD and psoriasis, although its effectiveness on asthmatic symptoms has been reported [26]. Here, we investigated whether Sal A administration ameliorated the development of AD-like skin lesions in 2,4-dinitrochlorobenzene (DNCB)-treated mice. The effects of Sal A were compared with those of dexamethasone (DEX), a steroidal anti-inflammatory drug commonly used to treat AD (eczema).

## 2. Materials and Methods

Sal A (PubChem ID 329825115, molecular weight 494.45, Cas No. 96574-01-5, ≥96% HPLC) and 2,4-dinitrochlorobenzene were purchased from Sigma-Aldrich (St. Louis, MO, USA).

### 2.1. Animals and Treatment

Seven-week-old male BALB/c mice were purchased from DBL (Seoul, Korea). Mice were housed in the laboratory animal facility at Kyung Hee University under conditions at 20∼24°C with a 12°h light-dark cycle and provided with standard laboratory chow and water *ad libitum* [27]. The animal experimental protocol was reviewed and approved by the Institutional Animal Care and Use Committee of Kyung Hee University (KHSASP-21-069). Mice were divided into five groups (*n* = 5 per group) after 2 weeks of acclimation: (1) vehicle control, (2) DNCB, (3) DNCB + 5 mg/kg Sal A, (4) DNCB + 10 mg/kg Sal A, and (5) DNCB + DEX [14]. Mice were sensitized by applying DNCB (1%, 150 *μ*l) dissolved in an acetone∶olive oil mixture (3∶1 vol/vol) on the ventral skin (day 0). Mice were challenged by applying DNCB (0.3%, 200 *μ*l) to both ears (10 *μ*l each) every other days (day 7–48). Sal A (5 or 10 mg/kg body weight) or DEX (DEX, 10 mg/kg) was administrated via intraperitoneal injection 30 min before challenge (day 19–47) [14]. All mice were sacrificed on day 49 (Figure 1). DEX was used as a positive control.

The article "Salvianolic Acid A Suppresses DNCB-Induced Atopic Dermatitis-Like Symptoms in BALB/c Mice" was published in 2021. Journal: Evid Based Complement Alternat Med.

### 2.2. Histological Examination

The ear skin of each mouse was prepared on day 49 to evaluate epidermal thickening. The ears from different experimental groups were fixed with neutral-buffered formalin (10%), dehydrated in sucrose solution (30%), and embedded in O.C.T. compound. We stained the sections with toluidine blue O or hematoxylin and eosin (H&E). Ear tissues from the five mice were examined in each group. We measured thickness of ears from the photographs of H&E-stained sections. The thickness was measured twice in five optical fields using a magnification of 200× and the mean value of each mouse was used.

### 2.3. IgE, Th2, Th1, and Th17 Cytokines

We collected serum on day 49 and stored at −80°C until use. We measured serum IgE levels by using an ELISA kit (eBioscience, San Diego, CA, USA) according to the manufacturer's instructions. The levels of Th2 cytokines (IL-4 and IL-13), Th17 cytokine (IL-17A), and Th1 cytokine (IFN-*γ*) were also measured in the ears and lymph nodes by reverse transcriptase polymerase chain reaction (RT-PCR). Synthesis of first-strand cDNA, specific primers, and PCR conditions were described as previously [28]. Aliquots (7 *μ*L) were electrophoresed in 1.2% agarose gels and stained with StaySafe^TM^ Nucleic Acid Gel Stain (Real Biotech Corporation, Taipei, Taiwan). We quantified the intensity of each PCR product using ImageJ software (NIH, Bethesda, MD, USA) and normalized to GAPDH levels [29].

### 2.4. Statistics

We performed statistical analysis with GraphPad Prism software (GraphPad Software, Inc., La Jolla, CA, USA). The data were expressed as means ± standard error of the mean (SEM). One-way analysis of variance (ANOVA) followed by Tukey's multiple comparison test was used for comparing differences among multiple groups. Differences were considered statistically significant at *p* < 0.05.

The article "Salvianolic Acid A Suppresses DNCB-Induced Atopic Dermatitis-Like Symptoms in BALB/c Mice" was published in 2021. Journal: Evid Based Complement Alternat Med.

## 3. Results

### 3.1. Sal A Ameliorated DNCB-Induced AD-Like Symptoms in BALB/C Mice

To investigate the effects of Sal A on AD-like symptoms in BALB/c mice, we sensitized and challenged skins with DNCB. Seven days after the sensitization, we treated mice with DNCB on both ears every other day (Figure 1). Sal A (5 or 10 mg/kg) or DEX (10 mg/kg) was delivered by intraperitoneal injection 30 min before the DNCB challenge from day 19 to evaluate its therapeutic potential for AD-like symptoms. On day 49, the ears of DNCB-treated BALB/c mice showed severe edema, erythema, erosion, dryness, and cracking of the skin (Figure 2(a)). Cotreatment of Sal A or DEX decreased severity of AD-like symptom (Figure 2(a)). We found that DNCB induced increased infiltration of immune cells in the H&E staining compared to the control group (Figure 2(b)). Furthermore, the epidermis was obviously thickened in the DNCB-treated group upon visual inspection due to hyperkeratosis (Figure 2(b)). DNCB treatment increased ear thickness in BALB/c mice (Figure 2(b)). The ears from DNCB-treated mice were swollen and showed epidermal hypertrophy (Figure 2(b)). The ears from Sal A (5 mg/kg and 10 mg/kg) or DEX (10 mg/kg)-treated mice, in contrast, exhibited less severe epidermal hypertrophy compared to those from DNCB-treated mice (Figure 2(b)). Treatment with Sal A or DEX attenuated markedly the increase of ear thickness by DNCB (Figure 2(c)). The efficacy of Sal A was similar to that of DEX, a well-known steroidal anti-inflammatory agent (Figures 2(b) and 2(c)).

### 3.2. Sal A Decreased DNCB-Induced Mast Cells Infiltration into the Skin Lesions in Mice

To investigate the effect of Sal A on mast cells infiltration into skin lesions in BALB/c mice, collected tissue sections were stained with toluidine blue O. The number of toluidine blue O-stained mast cells in skin lesions was significantly increased in the sections from DNCB-treated mice compared to those of control mice (Figure 3(a)). Treatment with Sal A or DEX significantly reduced the number of mast cells infiltrated in the ears from DNCB-treated mice (Figures 3(a) and 3(b)). The efficacy of Sal A was similar to that of DEX (Figures 3(a) and 3(b)).

### 3.3. Sal A Decreased DNCB-Induced Increases of Th2, Th1, and Th17 Cytokines in BALB/C Mice

Not only Th2 cells but also Th1/Th17 cells are suggested to be involved in AD [7, 30, 31]. Thus, we examined cytokine levels in ear skins. We measured the mRNA levels of the Th2 cytokines IL-4 and IL-13, the Th17 cytokine IL-17A, and the Th1 cytokine INF-*γ* in the ears. We found that the mRNA levels of Th2 cytokines IL-4 and IL-13 were significantly increased in skin lesions of DNCB-treated BALB/c mice compared with the control mice (Figures 4(a) and 4(b)). However, treatment with Sal A or DEX significantly decreased the level of Th2 cytokines IL-4 and IL-13 in the ear skin of DNCB-treated BALB/c mice (Figures 4(a) and 4(b)). The mRNA levels of Th17 cytokine IL-17 were also significantly increased in skin lesions from DNCB-treated mice compared to control mice (Figure 4(c)) and the levels of Th1 cytokine IFN-*γ* were also significantly increased in DNCB-treated mice compared to control mice (Figure 4(d)). However, treatment with Sal A or DEX significantly decreased the level of IL-17 and IFN-*γ* in the ear skin of DNCB-treated mice (Figures 4(c) and 4(d)).

The article "Salvianolic Acid A Suppresses DNCB-Induced Atopic Dermatitis-Like Symptoms in BALB/c Mice" was published in 2021. Journal: Evid Based Complement Alternat Med.

### 3.4. Sal A Decreased DNCB-Induced AD-Like Responses in Lymph Nodes

We found the enlarged cervical lymph nodes in DNCB-treated BALB/c mice compared with the control mice (Figures 5(a) and 5(b)). The DNCB-induced increase of lymph node weight was 1318% (Figure 5(b)). However, treatment with 10 mg/kg Sal A or DEX significantly decreased the sizes of lymph nodes from the DNCB-treated mice (Figures 5(a) and 5(b)). Sal A-induced decrease in lymph node weight was 22% (Figure 5(b)).

### 3.5. Sal A Suppressed DNCB-Induced Increases in Cytokine Levels in the Lymph Nodes

Similarly, the cytokine levels produced by Th2/Th17/Th1 cells in lymph nodes were investigated. The levels of cytokine mRNA were increased significantly in the cervical lymph nodes by repeated topical application of DNCB (Figure 6). Administration of Sal A decreased significantly the increases of IL-13, IL-17, and INF-*γ* levels (Figures 6(b)–6(d)), but not IL-4 level (Figure 6(a)). DEX treatment reduced DNCB-induced increases in the levels of IL-4, IL-13, and INF-*γ* (Figures 6(a), 6(b), and 6(d)), but not in IL-17 level (Figure 6(c)).

### 3.6. Sal A Decreased the DNCB-Induced Increase of Serum IgE Level in BALB/C Mice

Next, we investigated the effect of Sal A on DNCB-induced increase in serum IgE level in BALB/c mice. Serum IgE levels were significantly increased by repeated topical application of DNCB compared to control mice (Figure 7). However, treatment with Sal A or DEX significantly decreased the level of serum IgE (Figure 7).

## 4. Discussion

AD patients have common features with allergic asthma and rhinitis, that is, proinflammatory mediators from activated immune cells [32, 33]. Currently, immunosuppressive corticosteroids are used for AD treatment. However, corticosteroid use for long periods of time leads to severe side effects [34]. Therefore, finding novel natural chemicals from medicinal plants with fewer side effects should be performed to treat AD [34]. Various immune regulators from natural herbal extracts could have therapeutic potentials for AD [11–13]. Ethnopharmacologic studies on Radix Salviae suggest beneficial effects including anti-inflammation, antioxidant activity, and immune regulation.

The article "Salvianolic Acid A Suppresses DNCB-Induced Atopic Dermatitis-Like Symptoms in BALB/c Mice" was published in 2021. Journal: Evid Based Complement Alternat Med.

Previously, extracts from *S. miltiorrhiza* have shown immune regulatory effects on *Listeria* infection in Balb/c mice by decreasing serum IgE levels and IL-1*β* and by increasing natural killer (NK) cells, macrophages, and peripheral lymphocytes [35]. Among isolated natural chemicals from *S. miltiorrhiza*, cryptotanshinone and salvianolic acid B were found as the major components [22, 34]. Cryptotanshinone ameliorated secretion of TNF-*α* and IL-1*β*, infiltration of immune cells into skin lesions in DNCB-induced AD-like skin lesions in vivo and inhibited mast cell degranulation by IgE in vitro via inhibition of Syk and Lyn kinases [34]. Salvianolic acid B-containing microemulsion alleviated severity of imiquimod-induced psoriasis-like dermatitis, inhibited IL-23/IL-17 cytokines, reduced acanthosis, inhibited epidermal proliferation, and increased skin hydration [22]. In ovalbumin-induced asthmatic mice, tanshinone I and tanshinone IIA showed inhibitory effects on mast cell degranulation in RBL-2H3 mast cells and Sal A and tanshinone IIA showed significant inhibitory effects on features of allergic asthma in mice [26]. Daily administration of water or ethanolic extract of *S. miltiorrhiza* significantly reduced airway infiltration of inflammatory cells, Th1/Th2 cytokine levels, and goblet cell hyperplasia induced by ovalbumin [36]. However, effects of Sal A on AD development have not been studied.

Our results demonstrate that administration of Sal A attenuated DNCB-induced AD-like symptoms in BALB/c mice. Sal A treatment alleviated significantly disease severity and hypertrophy of ear skin and increased serum IgE levels. Furthermore, Sal A treatment decreased mast cells infiltration into skin lesions and lowered cytokine levels (IL-4, IL-13, IL-17, and IFN-*γ*) in DNCB-treated BALB/c mice. These effects of Sal A on skin lesions may be correlated with the Sal A effects on allergic asthma, because Th2 immune responses and infiltration of mast cells are cardinal features of both diseases [26]. In addition to cryptotanshinone, we elucidated that Sal A might be an active constituent for antiatopic pharmacology of *S. miltiorrhiza* [34].

In addition to the effects on ear skins, Sal A treatment reduced sizes of lymph nodes and cytokine levels in the lymph nodes. In the epidermis, DNCB exposure makes antigenic compounds and those antigens are engulfed by Langerhans cells, specialized dendritic cells in the skin. The antigen-recognizing Langerhans cells move to close lymph nodes and present the antigens to naïve T cells. Naïve T cells differentiate into Th2 cells, which secret IL-4, IL-5, and IL-13 in the early response and cooperate with Th1 cells and Th17 cells in the late response. Therefore, analyzing conditions of lymph nodes is an important parameter for the immune responses of atopic dermatitis. However, the effect of Sal A on lymph node sizes was smaller than that of DEX. On the other hand, the effect of Sal A on IL-17 levels in lymph nodes was greater than that of DEX. Differential effects of Sal A may imply unique ways of Sal A actions compared to DEX. Also, compounding results of Sal A on cytokine levels in ear skin and lymph nodes are needed to be confirmed at the protein levels in the future. These results from skin and lymph nodes may imply that Sal A administration could be helpful for the treatment of AD.

The article "Salvianolic Acid A Suppresses DNCB-Induced Atopic Dermatitis-Like Symptoms in BALB/c Mice" was published in 2021. Journal: Evid Based Complement Alternat Med.

Present results indicated that Sal A inhibits the development of AD-like skin lesions in BALB/c mice. Underlining mechanisms may be downregulation of proinflammatory cytokines, that is, Th2 (IL-4 and IL-13), Th17 (IL-17), and Th1 (IFN-*γ*)-associated factors, which resulted in inhibition of skin thickness, decrease of mast cells infiltration, and decrease of serum IgE production. The decrease of Th2 response factors, IL-4 and IL-13, plays a key role in the disease development. Especially, Th2-driven cytokines play important roles in the early phase of atopic eczema, such as eosinophils attraction, resulting in sequential activation of Th17- and Th1-type cells [37]. The essential roles of IL-4 and IL-13 in the pathogenesis of allergic diseases, such as AD and asthma, were proven clinically by the efficacy of dupilumab, a monoclonal antibody for IL-4R*α* [38, 39]. IL-4 and IL-13 are known to induce isotype switching to IgE synthesis by B cells, which results in activation of mast cells [40, 41]. IL-17 induces production of IL-4 from Th2 cells and differentiation of B cells to IgE-producing plasma cells [42–44]. Th1 response factor IFN-*γ* is also related with disease severity of AD [37, 45]. IFN-*γ* activates keratinocytes to express Fas (CD95), leading to apoptosis of keratinocytes and subsequent formation of eczematous lesions [45, 46]. Decrease in IFN-*γ* levels might contribute in the effects of Sal A in mice.

In previous studies, Sal A treatment resulted in downregulation of NF-*κ*B p65 expression [47–49]. Sal A showed inhibitory effects on not only Th2 cytokines but also Th1/Th17 cytokines, suggesting that the antiatopic activity of Sal A may originate from its anti-inflammatory effects. In line with these studies, the anti-inflammatory effects of Sal A may contribute to the antiatopic effects observed in the present study. In summary, Sal A regulates the immune response in the dermis, especially by suppressing the Th2/Th17/Th1 immune responses in a model of AD. Sal A showed antiatopic activity in a DNCB-induced mouse atopic dermatitis model, providing evidence for its therapeutic potential.

The article "Salvianolic Acid A Suppresses DNCB-Induced Atopic Dermatitis-Like Symptoms in BALB/c Mice" was published in 2021. Journal: Evid Based Complement Alternat Med.

## Figures and Tables

**Figure 1:** Experimental protocol: (A) BALB/c mice were divided into five groups: (1) vehicle control, (2) DNCB + vehicle, (3) DNCB + 5 mg/kg Sal A, (4) DNCB + 10 mg/kg Sal A, and (5) DNCB + DEX. To induce AD-like symptoms, DNCB was topically applied on BALB/c mice. DNCB (1%) was applied on day 0. After seven days, 0.3% DNCB was challenged every other days on the ears for the experiment (day 7–48). Sal A or DEX was administrated every other days starting from day 19 for 3 weeks (day 19–47). Mice were sacrificed on day 49.

**Figure 2:** Effect of Sal A on DNCB-induced AD-like lesions in BALB/c mice. (a) Photographed images of ears from each group were taken on day 49. (b) H&E-stained ear section on day 49 (400×). (c) Ear thickness was measured from the sections (*n* = 5). Data represent the mean ± SEM (*n* = 5). ^*∗∗∗*^*p* < 0.001 vs. the control group; ^###^*p* < 0.001 vs. the DNCB-treated group.

**Figure 3:** Effect of Sal A on DNCB-induced mast cell accumulation in skin lesions of BALB/c mice. (A) Representative images depicting the histological features of skin collected on day 49 are shown. Red arrows indicate mast cells. Toluidine blue O staining was used to identify mast cells. Cells were counted under a microscope at 400× magnification. The numbers of mast cells in the skin were calculated. Data represent the mean ± SEM (*n* = 5). ^*∗∗∗*^*p* < 0.001 vs. the control group; ^###^*p* < 0.001 vs. the DNCB-treated group.

**Figure 4:** Effect of Sal A on DNCB-induced increases in Th2, Th1, and Th17 cytokine levels in the ears. RT-PCR analyses for Th2 cytokines IL-4 (a) and IL-13 (b), Th17 cytokine IL-17A (c), and Th1 cytokine INF-*γ* (d). Results are presented as means ± SEM (*n* = 5). ^*∗∗∗*^*p* < 0.001 vs. the control group; ^#^*p* < 0.05, ^##^*p* < 0.01, ^###^*p* < 0.001 vs. the DNCB-treated group.

**Figure 5:** Effect of Sal A on the lymph nodes in DNCB-induced AD-like responses in mice. (a) Images of lymph nodes. (b) Weights of lymph nodes. ^*∗∗∗*^*p* < 0.001 vs. the control group; ^#^*p* < 0.05, ^###^*p* < 0.001 vs. the DNCB-treated group.

**Figure 6:** Effect of Sal A on the DNCB-induced increase in Th2, Th1, and Th17 cytokine levels in the lymph nodes. RT-PCR analyses for Th2 cytokines IL-4 (a) and IL-13 (b), Th17 cytokine IL-17A (c), and Th1 cytokine INF-*γ* (d). Results are presented as means ± SEM (*n* = 5). ^*∗∗∗*^*p* < 0.001 vs. the control group; ^#^*p* < 0.05, ^##^*p* < 0.01, ^###^*p* < 0.001 vs. the DNCB-treated group.

The article "Salvianolic Acid A Suppresses DNCB-Induced Atopic Dermatitis-Like Symptoms in BALB/c Mice" was published in 2021. Journal: Evid Based Complement Alternat Med.

**Figure 7:** Effect of Sal A on DNCB-induced increase in serum IgE level in BALB/c mice. Serum was collected on day 49. The level of serum IgE was measured with ELISA. Data are the means ± SEM (*n* = 5). ^*∗∗∗*^*p* < 0.001 vs. the control group; ^###^*p* < 0.001 vs. the DNCB-treated group.

## Data Availability

The data used to support the findings of this study are available from the corresponding author upon request.

## References

[1] Davidson W. F., Leung D. Y. M., Beck L. A. (2019). Report from the national institute of allergy and infectious diseases workshop on “atopic dermatitis and the atopic march: mechanisms and interventions”. *The Journal of Allergy and Clinical Immunology*.

[2] Leung D. Y., Guttman-Yassky E. (2017). Assessing the current treatment of atopic dermatitis: unmet needs. *The Journal of Allergy and Clinical Immunology*.

[3] Leung D. Y. M., Soter N. A. (2001). Cellular and immunologic mechanisms in atopic dermatitis. *Journal of the American Academy of Dermatology*.

[4] Vestergaard C., Yoneyama H., Murai M. (1999). Overproduction of Th2-specific chemokines in NC/Nga mice exhibiting atopic dermatitis–like lesions. *Journal of Clinical Investigation*.

[5] Spergel J. M., Mizoguchi E., Oettgen H., Bhan A. K., Geha R. S. (1999). Roles of T H 1 and T H 2 cytokines in a murine model of allergic dermatitis. *Journal of Clinical Investigation*.

[6] Chen L., Martinez O., Overbergh L., Mathieu C., Prabhakar B. S., Chan L. S. (2004). Early up‐regulation of Th2 cytokines and late surge of Th1 cytokines in an atopic dermatitis model. *Clinical and Experimental Immunology*.

[7] Koga C., Kabashima K., Shiraishi N., Kobayashi M., Tokura Y. (2008). Possible pathogenic role of Th17 cells for atopic dermatitis. *Journal of Investigative Dermatology*.

[8] Blume‐Peytavi U., Wahn U. (2011). Optimizing the treatment of atopic dermatitis in children: a review of the benefit/risk ratio of methylprednisolone aceponate. *Journal of the European Academy of Dermatology and Venereology*.

[9] Hengge U. R., Ruzicka T., Schwartz R. A., Cork M. J. (2006). Adverse effects of topical glucocorticosteroids. *Journal of the American Academy of Dermatology*.

[10] Jin H., He R., Oyoshi M., Geha R. S. (2009). Animal models of atopic dermatitis. *Journal of Investigative Dermatology*.

[11] Song H.-Y., Kim W. S., Mushtaq S. (2019). A novel chrysin derivative produced by gamma irradiation attenuates 2, 4-dinitrochlorobenzene-induced atopic dermatitis-like skin lesions in Balb/c mice. *Food and Chemical Toxicology*.

The article "Salvianolic Acid A Suppresses DNCB-Induced Atopic Dermatitis-Like Symptoms in BALB/c Mice" was published in 2021. Journal: Evid Based Complement Alternat Med.

[12] Ku J. M., Hong S. H., Kim S. R. (2018). The prevention of 2, 4-dinitrochlorobenzene-induced inflammation in atopic dermatitis-like skin lesions in BALB/c mice by Jawoongo. *BMC Complementary and Alternative Medicine*.

[13] Bai X.-Y., Liu P., Chai Y.-W. (2020). Artesunate attenuates 2, 4-dinitrochlorobenzene-induced atopic dermatitis by down-regulating Th17 cell responses in BALB/c mice. *European Journal of Pharmacology*.

[14] Kang J., Im D.-S. (2020). FFA2 activation ameliorates 2,4-dinitrochlorobenzene-induced atopic dermatitis in mice. *Biomolecules & Therapeutics*.

[15] Kang J., Lee J.-H., Im D.-S. (2020). Topical application of S1P(2) antagonist JTE-013 attenuates 2,4-dinitrochlorobenzene-induced atopic dermatitis in mice. *Biomolecules & Therapeutics*.

[16] Zhang E. Y., Chen A. Y., Zhu B. T. (2009). Mechanism of dinitrochlorobenzene-induced dermatitis in mice: role of specific antibodies in pathogenesis. *PLoS One*.

[17] Son S.-E., Park S.-J., Koh J.-M., Im D.-S. (2020). Free fatty acid receptor 4 (FFA4) activation ameliorates 2,4-dinitrochlorobenzene-induced atopic dermatitis by increasing regulatory T cells in mice. *Acta Pharmacologica Sinica*.

[18] Tse T. W. (2003). Use of common Chinese herbs in the treatment of psoriasis. *Clinical and Experimental Dermatology*.

[19] Boneberger S., Rupec R. A., Ruzicka T. (2010). Complementary therapy for atopic dermatitis and other allergic skin diseases: facts and controversies. *Clinics in Dermatology*.

[20] Fan Y., Luo Q., Wei J. (2018). Mechanism of salvianolic acid B neuroprotection against ischemia/reperfusion induced cerebral injury. *Brain Research*.

[21] Ma Z. G., Xia H. Q., Cui S. L., Yu J. (2017). Attenuation of renal ischemic reperfusion injury by salvianolic acid B via suppressing oxidative stress and inflammation through PI3K/Akt signaling pathway. *Brazilian Journal of Medical and Biological Research*.

[22] Guo J.-W., Cheng Y.-P., Liu C.-Y. (2020). Salvianolic acid B in microemulsion formulation provided sufficient hydration for dry skin and ameliorated the severity of imiquimod-induced psoriasis-like dermatitis in mice. *Pharmaceutics*.

[23] Wang S., Zhu L., Xu Y., Qin Z., Xu A. (2020). Salvianolic acid B ameliorates psoriatic changes in imiquimod-induced psoriasis on BALB/c mice by inhibiting inflammatory and keratin markers via altering phosphatidylinositol-3-kinase/protein kinase B signaling pathway. *The Korean Journal of Physiology & Pharmacology*.

[24] Kim H.-M., Lee E.-H., Lee J.-H., Jung J.-A., Kim J.-J. (1999). Salviae radix root extract inhibits immunoglobulin E-mediated. *General Pharmacology: The Vascular System*.

[25] Trinh H. T., Chae S. J., Joh E.-H., Son K. H., Jeon S. J., Kim D.-H. (2010). Tanshinones isolated from the rhizome of Salvia miltiorrhiza inhibit passive cutaneous anaphylaxis reaction in mice. *Journal of Ethnopharmacology*.

The article "Salvianolic Acid A Suppresses DNCB-Induced Atopic Dermatitis-Like Symptoms in BALB/c Mice" was published in 2021. Journal: Evid Based Complement Alternat Med.

[26] Heo J.-Y., Im D.-S. (2019). Anti-allergic effects of salvianolic acid A and tanshinone IIA from Salvia miltiorrhiza determined using in vivo and in vitro experiments. *International Immunopharmacology*.

[27] Huang J., Su M., Lee B.-K., Kim M.-J., Jung J. H., Im D.-S. (2018). Suppressive effect of 4-hydroxy-2-(4-hydroxyphenethyl) isoindoline-1,3-dione on ovalbumin-induced allergic asthma. *Biomolecules & Therapeutics*.

[28] Park S. J., Im D. S. (2019). Blockage of sphingosine-1-phosphate receptor 2 attenuates allergic asthma in mice. *British Journal of Pharmacology*.

[29] Lee J.-M., Park S.-J., Im D.-S. (2017). Calcium signaling of lysophosphatidylethanolamine through LPA1 in human SH-SY5Y neuroblastoma cells. *Biomolecules & Therapeutics*.

[30] Kim J.-Y., Jeong M. S., Park M. K., Lee M.-K., Seo S. J. (2014). Time-dependent progression from the acute to chronic phases in atopic dermatitis induced by epicutaneous allergen stimulation in NC/Nga mice. *Experimental Dermatology*.

[31] Muraro A., Lemanske R. F., Hellings P. W. (2016). Precision medicine in patients with allergic diseases: airway diseases and atopic dermatitis-PRACTALL document of the European academy of allergy and clinical immunology and the American academy of allergy, asthma & immunology. *The Journal of Allergy and Clinical Immunology*.

[32] Bantz S. K., Zhu Z., Zheng T. (2014). The atopic march: progression from atopic dermatitis to allergic rhinitis and asthma. *Journal of Clinical & Cellular Immunology*.

[33] Akdis C. A., Akdis M., Bieber T. (2006). Diagnosis and treatment of atopic dermatitis in children and adults: European academy of allergology and clinical immunology/American academy of allergy, asthma and immunology/PRACTALL consensus report. *The Journal of Allergy and Clinical Immunology*.

[34] Buyanravjikh S., Han S., Lee S. (2018). Cryptotanshinone inhibits IgE-mediated degranulation through inhibition of spleen tyrosine kinase and tyrosine-protein kinase phosphorylation in mast cells. *Molecular Medicine Reports*.

[35] Gao D., Mendoza A., Lu S., Lawrence D. A. (2012). Immunomodulatory effects of danshen (Salvia miltiorrhiza) in BALB/c mice. *ISRN Inflamm*.

[36] Luo J., Zhang L., Zhang X. (2019). Protective effects and active ingredients of Salvia miltiorrhiza Bunge extracts on airway responsiveness, inflammation and remodeling in mice with ovalbumin-induced allergic asthma. *Phytomedicine*.

[37] Grewe M., Bruijnzeel-Koomen C. A. F. M., Schöpf E. (1998). A role for Th1 and Th2 cells in the immunopathogenesis of atopic dermatitis. *Immunology Today*.

The article "Salvianolic Acid A Suppresses DNCB-Induced Atopic Dermatitis-Like Symptoms in BALB/c Mice" was published in 2021. Journal: Evid Based Complement Alternat Med.

[38] Gandhi N. A., Pirozzi G., Graham N. M. H. (2017). Commonality of the IL-4/IL-13 pathway in atopic diseases. *Expert Review of Clinical Immunology*.

[39] Wenzel S., Ford L., Pearlman D. (2013). Dupilumab in persistent asthma with elevated eosinophil levels. *New England Journal of Medicine*.

[40] Leung D. Y. M., Boguniewicz M., Howell M. D., Nomura I., Hamid Q. A. (2004). New insights into atopic dermatitis. *Journal of Clinical Investigation*.

[41] Williams C. M. M., Galli S. J. (2000). Mast cells can amplify airway reactivity and features of chronic inflammation in an asthma model in mice. *Journal of Experimental Medicine*.

[42] Sugaya M. (2020). The role of Th17-related cytokines in atopic dermatitis. *International Journal of Molecular Sciences*.

[43] Nakajima S., Kitoh A., Egawa G. (2014). IL-17A as an inducer for Th2 immune responses in murine atopic dermatitis models. *Journal of Investigative Dermatology*.

[44] Milovanovic M., Drozdenko G., Weise C., Babina M., Worm M. (2010). Interleukin-17A promotes IgE production in human B cells. *Journal of Investigative Dermatology*.

[45] Ong P. Y., Leung D. M. Y. (2006). Immune dysregulation in atopic dermatitis. *Current Allergy and Asthma Reports*.

[46] Trautmann A., Akdis M., Kleemann D. (2000). T cell–mediated Fas-induced keratinocyte apoptosis plays a key pathogenetic role in eczematous dermatitis. *Journal of Clinical Investigation*.

[47] Zhang W., Song J.-K., Zhang X. (2018). Salvianolic acid A attenuates ischemia reperfusion induced rat brain damage by protecting the blood brain barrier through MMP-9 inhibition and anti-inflammation. *Chinese Journal of Natural Medicines*.

[48] Fan H.-Y., Yang M.-Y., Qi D. (2015). Salvianolic acid A as a multifunctional agent ameliorates doxorubicin-induced nephropathy in rats. *Scientific Reports*.

[49] Yuan X., Xiang Y., Zhu N. (2017). Salvianolic acid A protects against myocardial ischemia/reperfusion injury by reducing platelet activation and inflammation. *Experimental and Therapeutic Medicine*.

